This article has been retracted.

# LINC00707 Promotes Cell Proliferation in Cervical Cancer via the miR-374c-5p/SDC4 Axis

**DOI:** 10.1155/2022/5793912

**Published:** 2022-07-28

**Authors:** Fang Fang, Chunfeng Guo, Weinan Zheng, Qingyang Li

**Affiliations:** ^1^Department of Obstetric and Gynecology, Renmin Hospital of Wuhan University, Wuhan 430000, China; ^2^Department of Gynecology, The First Affiliated Hospital of Xinjiang Medical University, Urumchi 830001, China; ^3^Department of Human Anatomy and Embryology, Chengdu Medical College, Chengdu 610000, China; ^4^Department of Gynecology and Obstetrics, Xinjiang Production and Construction Corps 13 Division Red Star Hospital, Hami City 839000, China

## Abstract

Cervical cancer (CC) is the second main reason of cancer-related deaths in women around the world. Long intergenic nonprotein coding RNA 707, which is known as LINC00707, has been elucidated to facilitate the progression of multifarious tumors, but how it may exert functions in CC has not been elucidated yet. By using quantitative real-time RT-PCR (RT-qPCR), we identified the expression pattern LINC00707 may possess in CC. Loss-of-function assays including Cell Counting Kit-8 (CCK-8), colony formation, and transferase-mediated dUTP nick-end labeling (TUNEL) assays were taken to verify the effects of LINC00707 inhibition on CC cell proliferation and apoptosis. The downstream RNAs were selected through bioinformatics prediction, and their interaction with LINC00707 was verified through mechanism assays including the luciferase reporter assay, RNA pull-down assay, and RNA immunoprecipitation (RIP) assay. According to results, LINC00707 was upregulated in CC cells, and LINC00707 insufficiency inhibited cell proliferation while facilitating cell apoptosis. MicroRNA (miRNA) miR-374c-5p interacted with LINC00707, and syndecan-4 (SDC4) was verified to be the downstream target gene. Data of rescue assays proved that LINC00707 could promote CC cell malignancy via the miR-374c-5p/SDC4 axis, which revealed a potential treatment option for CC.

## 1. Introduction

Cervical cancer (CC) is one of the most familiar malignant tumors in the female genital system, resulting in a great deal of cancer-related deaths globally, especially in underdeveloped and developing countries [1]. In spite of great progress made in methods of diagnosis and treatment for CC [2], the overall outcomes remain unsatisfying. Hence, it is of necessity to clarify the molecular mechanism beneath CC progression so as to recognize and offer more effective diagnostic biomarkers and therapeutic targets for medical treatment of CC.

As crucial regulators, long noncoding RNAs (lncRNAs) exert considerable roles in numerous cancers by influencing many cellular processes, regulating gene expression during different stages of cancer development [3]. lncRNA-Hh promotes the generation of cancer stem cells in breast cancer by activating the hedgehog signaling pathway [4]. lncRNA LINC01207 facilitates cell proliferation in lung adenocarcinoma [5]. lncRNA MALAT1 with its upregulation in esophageal squamous cell carcinoma aggravates cell growth [6]. LINC00707 has been illustrated to possess carcinogenic property in cancers. It accelerates the proliferation along with metastasis of lung adenocarcinoma by upregulating Cdc42 [7]. It is determined to accelerate breast cancer via the modulation of the miR-30c/CTHRC1 loop [8]. Combined with these considerations, we are interested in LINC00707 and we try to verify how LINC00707 may exert certain impacts on CC.

In this study, we planned to figure out what specific impacts LINC00707 may exert on CC progression, and we found that LINC00707 promoted cell proliferation in CC via the miR-374c-5p/SDC4 axis, which may provide new thoughts for treating CC.

## 2. Materials and Methods

### 2.1. Cell Culture

Human cervical epithelial immortalized cell line (H8), along with CC cell lines (SiHa, HeLa, CaSki, and C-33A), was purchased from the Chinese Academy of Sciences (Beijing, China). They were incubated in Dulbecco's modified Eagle medium (DMEM) (Gibco-BRL, Grand Island, NY, USA) which contained 10% fetal bovine serum (FBS) (Gibco-BRL) plus 100 mg/mL penicillin and streptomycin (Invitrogen, Carlsbad, CA, USA). The condition for cell cultivation was set as 5% CO_2_ at 37°C in a humid atmosphere.

### 2.2. Cell Transfection

After transfection of 48 h, SiHa and HeLa cells were put into 6-well plates at a cell density of 70%-80%. shRNAs against LINC00707 (sh-LINC00707#1/2) and SDC4 (sh-SDC4#1/2), along with their negative controls (shNCs), were constructed to knock down LINC00707 or SDC4 expression. The miR-374c-5p mimics, NC mimics, miR-374c-5p inhibitor, and NC inhibitor were all obtained from GeneChem (Shanghai, China) for the overexpression or silencing of miR-374c-5p in CC cells. The above control plasmids were transfected with Lipofectamine (Invitrogen, Carlsbad, CA, USA).

### 2.3. Quantitative Real-Time RT-PCR

By using the TRIzol reagent (Invitrogen, Carlsbad, USA), we supplemented the extraction of total RNA from CC cells, which were then reversely transcribed into cDNA by using the Reverse Transcription Kit (Invitrogen). RT-qPCR was processed on the Bio-Rad CFX96 system using the SYBR-Green Real-Time PCR Kit (Takara Bio Inc., Tokyo, Japan). The normalization was set as GAPDH or U6, with expression fold changes calculated by 2^−ΔΔCt^ methods. Each experiment went through three repeats.

### 2.4. Cell Viability Assay

SiHa and HeLa cells were planted in 96-well plates (Corning Costar, Corning, NY, USA), with a density of 1 × 10^3^ cells in each well, and then, they were cultured at five time points over 0, 24, 48, 72, and 96 h. 10 *μ*l of CCK-8 solution was added, and the cells were cultured for another 4 h. The absorbance at 450 nm was finally detected using the ELX-800 spectrometer reader (Bio-Tek Instruments Inc., Waltham, MA, USA).

### 2.5. TUNEL (Terminal Deoxynucleotidyl Transferase-Mediated Nick-End Labeling) Assay

In Situ Cell Death Detection Kit (Roche, Mannheim, Germany) was applied to evaluate cell apoptosis by the TUNEL staining assay based upon the standardized guidelines. DAPI (Haoran Biotechnology, Shanghai, China) or merge (Gene-denovo, Guangzhou, Guangdong, China) was employed for dyeing SiHa and HeLa cells. By using an EVOS FL microscope (Thermo Fisher Scientific, Massachusetts), relative fluorescence intensity was measured, and the calculation for cells was made using ImageJ software.

### 2.6. Western Bolt

Protein extraction reagent (Pierce, IL, USA) was used to obtain total protein. Proteins were isolated by 10% SDS-PAGE (Boster Biological Technology, LA, CA, USA) and then transferred to PVDF (East Fluorine Chemical Technology, Shanghai, China) after separation and blocked with milk. The membranes were incubated with specific antibodies: anti-Bcl-2 (ab32124, Abcam, Cambridge, UK), anti-Bax (ab32503, Abcam), anti-SDC4 (ab213830, Abcam), or GAPDH (ab8245, Abcam) which served as the internal reference. The amount of protein was detected by the chemiluminescence system (GE Healthcare, Chicago, IL, USA).

### 2.7. Luciferase Reporter Assay

The LINC00707 sequences or 3′-UTR fragments of SDC4 containing corresponding binding sites of miR-374c-5p were subcloned into the pmirGLO dual-luciferase vector (Promega), thereby constructing LINC00707/SDC4-WT, together with the corresponding mutant-type vector LINC00707/SDC4-MUT. Then, the plasmids were subjected to cotransfection with NC mimics or miR-374c-5p mimics into SiHa or HeLa cells. After 48 h of transfection, the luciferase activity was measured via the dual-luciferase reporter assay kit (Promega, USA) as per the guides of the manufacturer.

### 2.8. Colony Formation Assay

After transfection, 800-1000 cells were planted in 6-well plates. The medium was changed every 3 days, as required. Two weeks later, the cells were washed with PBS (Solibao Technology, Beijing, China) for two times. Methanol (Solarbio) was used for cell fixation for 15 minutes, and crystal violet (Beyotime Biotechnology, Nantong, China) was applied to dye the cells. Later, the visible colony numbers were counted using ImageJ software.

### 2.9. Subcellular Fractionation

The extracts of the cytoplasmic and nuclear component were gained from SiHa and HeLa cells with NE-PER Nuclear and Cytoplasmic Extraction Reagents (Thermo Scientific, Waltham, MA, USA). The cell cytoplasm was isolated by adding the cell fractionation buffer, and cell disruption buffer was used to collect the cell nucleus. At last, the content of LINC00707, as well as the cytoplasmic control GAPDH and the nucleus control U6, was presented.

### 2.10. RNA Pull-Down Assay

LINC00707-WT/Mut and miR-374c-5p-WT/Mut, along with the negative control NC, were biotinylated into Bio-LINC00707-WT/Mut, Bio-miR-374c-5p-WT/Mut, and Bio-NC. Then, the biotinylated RNA was cultured with cell lysate overnight. RNA-bound beads were cocultivated for 48 h, and finally, the purified RNA complexes were evaluated by RT-qPCR.

### 2.11. RIP Assay

This assay was conducted using Magna RNA-binding protein immunoprecipitation kit (Millipore, Billerica, MA, USA). Lysates of CC cells (SiHa and HeLa) were cultured in RIP buffer containing magnetic beads which were combined with the Ago2 antibody, with normal IgG regarded as the control. Finally, RNAs after purification were analyzed by RT-qPCR.

### 2.12. Statistical Analysis

For this study, every experiment went through three repeats. Represented as means ± standard deviation (SD), related data were subjected to analyses by the GraphPad Prism 7 software package (GraphPad Software, Inc., La Jolla, CA, USA). ANOVA and Student's *t*-test were applied to compare the difference of multiple groups and two groups. Data with statistical significance was set as *P* value below 0.05.

## 3. Results

### 3.1. Knockdown of LINC00707 Inhibits CC Cell Proliferation

At first, LINC00707 was examined to be with higher expression in CC cell lines (SiHa, HeLa, CaSki, and C-33A) than in the normal cell line (H8) (Figure 1(a)). Sh-LINC00707#1/2 was transfected into SiHa and HeLa cell lines that contained the highest LINC00707 expression to knock down its expression (Figure 1(b)), and LINC00707#1 with better efficiency was used for the next-step loss-of-function assays. After LINC00707 inhibition, SiHa and HeLa cells displayed weakened viability (Figure 1(c)). Validated by the reduced number of colonies in LINC00707-downregulated SiHa and HeLa cells, we could say that LINC00707#1 knockdown repressed cell proliferation (Figure 1(d)). Next, TUNEL data exhibited that absence of LINC00707 enhanced the apoptosis of CC cells (Figure 1(e)). Additionally, Bcl-2 protein expression was declined while Bax expression was elevated by LINC00707#1 shortage, indicating that LINC00707 inhibition facilitated cell apoptosis (Figure 1(f)).

### 3.2. LINC00707 Sponges miR-374c-5p in CC Cells

We carried out subcellular fractionation analysis to identify the cellular localization of LINC00707 in CC cells, and the majority cytoplasmic existence of LINC00707 was seen (Figure 2(a)). Cytoplasmic lncRNAs are well known as competing endogenous RNAs, namely, ceRNAs in cancer progression [9]. By using the online software program miRBase, we screened out 8 miRNAs (miR-376c-3p, miR-30c-5p, miR-30a-5p, miR-30d-5p, miR-30b-5p, miR-30e-5p, miR-374c-5p, and miR-338-3p) that have complementary base pairing with LINC00707 (Figure 2(b)). As shown by RNA pull-down data, miR-374c-5p presented the highest enrichment in the Bio-LINC00707-WT group (Figure 2(c)), so it was chosen for further investigations. The low expression of miR-374c-5p was verified in CC cell lines via RT-qPCR (Figure 2(d)). The binding sites between LINC00707 and miR-374c-5p were predicted by using a bioinformatics tool (Figure 2(e)). After miR-374c-5p overexpression, the LINC00707-WT group exhibited declined luciferase activity, with bare variation in the mutant group (Figure 2(f)). Finally, RT-qPCR data manifested that LINC00707 knockdown led to elevated miR-374c-5p expression (Figure 2(g)).

### 3.3. SDC4 Is Targeted by miR-374c-5p

As shown in Figure 3(a), SDC4 and ARID4A were predicted to combine with miR-374c-5p by starBase, making them potential downstream targets of miR-374c-5p. It was then verified through the RNA pull-down assay that SDC4 and ARID4A were both enriched in the Bio-miR-374c-5p-Wt group, while the enrichment of SDC4 was greater than that of ARID4A (Figure 3(b)). It was found by RT-qPCR analysis that SDC4 possessed a high expression pattern in CC cell lines (Figure 3(c)). What is more, LINC00707, SDC4, and miR-374c-5p exhibited high enrichment in the Ago2 antibody, which indicated their coexistence in RISC (RNA-induced silencing complex) (Figure 3(d)). To probe the interactions between miR-374c-5p and SDC4, we upregulated miR-374c-5p expression in the SiHa cell line via miR-374c-5p mimic transfection and inhibited its expression in C-33A cells by miR-374c-5p inhibitor transfection (Figure 3(e)). SDC4 was negatively regulated by miR-374c-5p, as evidenced via RT-qPCR along with western blot (Figure 3(f)). Furthermore, the binding sites of miR-374c-5p and SDC4 were conjectured by bioinformatics, and it was verified that the SDC4-WT group presented declined luciferase activity in miR-374c-5p mimic-transfected CC cells (Figure 3(g)). Furthermore, RT-qPCR data validated that SDC4 expression was declined by LINC00707 inhibition in CC cells (Figure 3(h)).

### 3.4. LINC00707 Promotes CC Cell Proliferation via the miR-374c-5p/SDC4 Axis

SDC4 expression was silenced in SiHa cells via sh-SDC4#1/#2 transfection (Figure 4(a)) for the follow-up rescue assays. The viability and proliferation of SiHa cells were suppressed by LINC00707 knockdown, while they were promoted upon the cotransfection of the miR-374c-5p inhibitor. Such effect was normalized again by the cotransfection of sh-SDC4#1 (Figures 4(b) and 4(c)). As for CC cell apoptosis, it was verified through the TUNEL assay that miR-374c-5p downregulation reversed the promoting effects of sh-LINC00707#1 on cell apoptosis, while this impact was normalized again by knockdown of SDC4 (Figure 4(d)). Same results were observed through western blot analysis (Figure 4(e)). In conclusion, LINC00707 promotes CC cell proliferation via the miR-374c-5p/SDC4 axis.

## 4. Discussion

Cervical cancer (CC) is one of the most common malignant cancers in females [10, 11]. Referring to concerned statistics, nearly 530,000 new cases are diagnosed universally each year [12], and the number of CC-caused mortality in low- and middle-income countries is remarkably higher than that in high-income countries [13]. Long noncoding RNAs (lncRNAs) are extensively linked with all kinds of cancer-related biological activities [14, 15]. Dysregulation of lncRNAs, together with their various impacts in CC, has been well elucidated [16, 17]. For example, lncRNA PVT1 accelerates cervical cancer progression by downregulating miR-424 [18]. lncRNA HOXA11 antisense aggravates tumor development and stemness maintenance in cervical cancer [19]. lncRNA HOXD-AS1 modulates cell proliferation in cervical cancer by motivating the Ras/ERK signaling pathway [20]. It has been documented that LINC00707 aggravates the development of many cancers, including colorectal cancer [21], osteosarcoma [22], and gliomas [23]. We verified the high expression of LINC00707 in CC for the first time, and we further validated that LINC00707 inhibition suppressed the malignant cell behaviors in CC.

lncRNAs are extensively affirmed to be the “sponge” or “ceRNA (competing endogenous RNA)” in the regulatory network involving with lncRNA, miRNA, and target genes [24]. For illustration, lncRNA HOTAIR exerts accelerating impact in gastric cancer malignancy via effectively becoming a sink for miR-331-3p and thus regulating the depression of HER2 [25]. lncRNA LINC00511 promotes tumorigenesis and stemness of breast cancer through regulating the signaling composed of miR-185-3p, E2F1, and Nanog [26]. lncRNA 00152 acts as a ceRNA to regulate NRP1 expression via sponging miRNA-206 in colorectal cancer [27]. By conducting subcellular localization analysis, the majority of LINC00707 in the cytoplasm of CC cells was observed, which suggested the potential ceRNA model. Through bioinformatics prediction along with related mechanism assays, miR-374c-5p was identified as the target of LINC00707, and SDC4 was further confirmed to be the downstream gene, which constituted a ceRNA model in CC cells. Results of rescue assays testified that LINC00707 could promote the malignant development of CC cells via sponging miR-374c-5p to elevate SDC4 expression. LINC00707 has been demonstrated to be involved in the ceRNA network to affect cancer progression such as hepatocellular carcinoma and colorectal cancer [21, 28], but it was the first time that we revealed a ceRNA pathway of LINC00707/miR-374c-5p/SDC4 in the regulation of CC cells. miR-374c-5p has been illustrated to regulate the invasion and migration of CC [29], and what we had discovered about miR-374c-5p in CC cell malignancy may help to provide more therapeutic strategies for CC treatment in the future.

To sum up, we confirmed through this research that LINC00707 promoted CC malignancy cells via the miR-374c-5p/SDC4 axis. Though the clinical significance of LINC00707 along with its regulatory mechanism remains to be verified in the future researches, we hope that our experimental outcomes can help shed some light on the future treatment for CC.

## Figures and Tables

**Figure 1:** LINC00707 knockdown inhibits CC cell proliferation. (a) LINC00707 expression in four CC cell lines (SiHa, HeLa, CaSki, and C-33A) and normal H8 cell line. (b) LINC00707 expression was knocked down in CC cells. (c, d) The effects of LINC00707#1 depletion on cell proliferation were validated by CCK-8 and colony formation assays. (e, f) The effects of LINC00707#1 depletion on cell apoptosis level were measured by TUNEL assay and western blot, with GAPDH as an internal control. Error bars represent the mean ± SD of at least three independent experiments. ^∗^*P* < 0.05, ^∗∗^*P* < 0.01.

**Figure 2:** LINC00707 sponges miR-374c-5p in CC cells. (a) LINC00707 localization identified by subcellular fractionation detection, with GAPDH and U6 as internal controls. (b) Potential miRNAs of LINC00707 predicted through starBase. (c) RNA pull-down assay was taken to detect the enrichment of the selected miRNA candidates in the Bio-LINC00707-WT group. (d) miR-374c-5p expression in CC cell lines was verified. (e) The binding sites between LINC00707 and miR-374c-5p were exhibited. (f) The luciferase activity of CC cells in LINC00707-WT and LINC00707-Mut groups upon miR-374c-5p mimic transfection. (g) miR-374c-5p expression in sh-LINC00707#1-transfected CC cells. Error bars represent the mean ± SD of at least three independent experiments. ^∗^*P* < 0.05, ^∗∗^*P* < 0.01.

**Figure 3:** SDC4 is the target gene of miR-374c-5p in CC cells. (a) Potential mRNAs that may bind to miR-374c-5p were selected using starBase. (b) RNA pull-down assay was taken to measure the enrichment of selected two mRNAs (SDC4 and ARID4A) in Bio-miR-374c-5p-WT/Mut groups. (c) The identified SDC4 expression in CC cell lines. (d) RIP assay was performed to test the enrichment of LINC00707, miR-374c-5p, and SDC4 in the anti-Ago2 group and the control IgG group. (e) miR-374c-5p expression was elevated in the SiHa cell line via miR-374c-5p mimic transfection while it was reduced via miR-374c-5p inhibitor transfection in C-33A cells. (f) The relative expression along with protein level of SDC4 upon miR-374c-5p overexpression or inhibition. (g) The binding sites between miR-374c-5p and SDC4 were evidenced by the luciferase reporter assay. (h) SDC4 expression in sh-LINC00707#1-transfected CC cells. Error bars represent the mean ± SD of at least three independent experiments. ^∗^*P* < 0.05, ^∗∗^*P* < 0.01, and ^∗∗∗^*P* < 0.001.

**Figure 4:** LINC00707 promotes CC cell proliferation via the miR-374c-5p/SDC4 axis. (a) Sh-SDC4#1/#2 transfection in the SiHa cell line to knock down gene expression. (b, c) The viability and proliferation of CC cells were measured by CCK-8 along with colony formation assay in different groups (sh-NC, sh-LINC00707#1, sh-LINC00707#1+miR-374c-5p inhibitor, and sh-LINC00707#1+miR-374c-5p inhibitor+sh-SDC4#1). (d, e) Cell apoptosis change was measured by TUNEL and western blot assays. GAPDH was an internal control. Error bars represent the mean ± SD of at least three independent experiments. ^∗^*P* < 0.05, ^∗∗^*P* < 0.01.

## Data Availability

The data used to support the findings of this study are included within the article.
